RETRACTED

# Effects of Pulmonary Surfactant Combined with Noninvasive Positive Pressure Ventilation on KRT-14 and ET-1 Levels in Peripheral Blood and Therapeutic Effects in Neonates with Respiratory Distress Syndrome

**DOI:** 10.1155/2021/4117800

**Published:** 2021-10-31

**Authors:** Lihan Huang, Hong Liang, Longbin Liu, Yucong Lin, Xinzhu Lin

**Affiliations:** ^1^Department of Neonatology, Women and Children's Hospital, School of Medicine, Xiamen University, Xiamen 361003, China; ^2^Xiamen Key Laboratory of Perinatal-Neonatal Infection, Xiamen, 361003 Fujian Province, China

## Abstract

This study is aimed at exploring the effect of pulmonary surfactant (PS) combined with noninvasive positive pressure ventilation on the levels of Keratin-14 (KRT-14) and Endothelin-1 (ET-1) in peripheral blood and the therapeutic effect of neonatal respiratory distress syndrome (NRDS). Altogether 137 cases of neonates with respiratory distress syndrome treated in our hospital from April 2016 to July 2018 were collected. Among them, 64 cases treated with noninvasive positive pressure ventilation were considered as the control group, and 73 cases treated with PS combined with noninvasive positive pressure ventilation were considered as the observation group. The expression of KRT-14 and ET-1 in the two groups was compared. The therapeutic effect, death, complications, and blood gas indexes PaO_2_, PaCO_2_, and PaO_2_/FiO_2_ in the two groups were compared. Receiver operating characteristic curve (ROC) was applied to analyze the diagnostic value of KRT-14 and ET-1 in the therapeutic effect of NRDS. The effective rate of the observation group was higher than that of the control group. After treatment, PaO_2_ and PaO_2_/FiO_2_ in both groups were notably higher than that before treatment, while PaCO_2_ was notably lower than that before treatment. And after treatment, the levels of PaO_2_ and PaO_2_/FiO_2_ in the observation group were remarkably higher than that in the control group; PaCO_2_ was notably lower than that in the control group. After treatment, the levels of KRT-14 and ET-1 in the two groups were remarkably lower than those before treatment, and the levels of KRT-14 and ET-1 in the observation group were considerably lower than those in the control group after treatment. ROC curve showed that the area under the curve (AUC) of KRT-14 was 0.791, and the AUC of ET-1 was 0.816. PS combined with noninvasive positive pressure ventilation can notably improve the therapeutic effect of NRDS. KRT-14 and ET-1 levels may be potential therapeutic diagnostic indicators.

## 1. Introduction

Neonatal respiratory distress syndrome (NRDS) is one of the most common diseases in neonatal intensive care unit, the incidence rate of which is about 7% among infants, and it is also one of the main causes of neonatal death in hospital in China [1, 2]. The main mechanism of the disease is hypoxemia and hypercapnia caused by lack of surfactant. The diffusion efficiency of oxygen through the alveolar-capillary exchange barrier is disturbed due to various factors, and lung injury in neonates will lead to asthma, septicemia, pneumonia, and other complicated symptoms [3]. Premature delivery of pregnant women and pregnancy diseases may lead to morbidity. Only early diagnosis and treatment can improve the quality of life of neonates [4, 5].

RETRACTED

Since the pathogenesis of NRDS is the lack of pulmonary surfactant, exogenous pulmonary surfactant (PS) replacement therapy is also found to be an effective treatment [6]. When neonates suffer from respiratory failure, respiratory support for them can also improve their condition. But invasive ventilation is easy to cause a series of complications such as lung infection, ventilator-associated lung injury, etc., which makes people pay wide attention to the clinical application of noninvasive ventilation [7]. It has been found in lots of studies that noninvasive positive pressure ventilation can significantly improve the condition of NRDS neonates and has good safety [8, 9]. At the same time, some studies also reveal that PS combined with noninvasive positive pressure ventilation can further improve the clinical efficacy [10].

Keratin-14 (KRT-14) is a cytoskeleton protein that has good diagnostic value for lung tissue injury [11]. A study by team of Confalonieri et al. [12] reported that KRT14 is a viable biomarker for activation and repair/regeneration of lung cells. It participates in the repair and regeneration of alveoli, and the alveoli collapsed, and lung cells were severely damaged in neonates with NRDS, so KRT14 may be used as an indicator of the improvement of the condition of neonates with RDS. Endothelin-1 (ET-1) is a vasoactive substance, which is mainly produced in lung tissue. It promotes the gradual change of pulmonary vascular reactivity through angiogenesis. It involves vascular regulation, bronchoconstriction, and inflammatory reaction in respiratory system. Endothelium and epithelial dysfunction in RDS patients can be caused by induction of proinflammatory mechanism. The use of endothelin receptor antagonist can regulate lung injury [13, 14]. The study of El's team [15] examined the plasma ET-1 concentration of 69 premature neonates aged 28 weeks to 34 weeks and diagnosed with NRDS. It is found that the ET-1 concentration on the 3rd day of birth increases significantly, and it has predictive value for whether the infant would develop bronchopulmonary dysplasia. At present, there is little research on the correlation of KRT-14 and ET-1 with curative effect of NRDS neonates.

RETRACTED

Therefore, this study is aimed at providing the basis and direction for clinical research through PS combined with noninvasive positive pressure ventilation to treat NRDS neonates and observing the levels of KRT-14 and ET-1 in peripheral blood.

## 2. Materials and Methods

Totally 137 neonates with NRDS treated in our hospital from April 2016 to July 2018 were collected. All neonates were admitted to hospital for basic treatment such as keeping breathing smooth, anti-infection, and maintaining water and electrolyte balance. Among them, 64 infants were included in the control group, who received treatment of noninvasive positive pressure ventilation on the basis of basic treatment, including 37 males and 27 females. The other 73 infants received treatment of PS combined with noninvasive positive pressure ventilation on the basis of basic treatment were considered as the observation group, including 38 males and 35 females. The study was approved by the Medical Ethics Committee, and all parents of the infants were informed and signed the informed consent form.

### 2.1. Inclusion and Exclusion Criteria

For inclusion criteria, all neonates were diagnosed as NRDS by imaging, and the diagnostic criteria were based on the European consensus guidelines on the management of respiratory distress syndrome-2016 update [16]. Newborns with complete clinical data and treatment.

For exclusion criteria, neonates had congenital immune defects. Neonates complicated with other respiratory diseases, acute infectious diseases, or liver and kidney insufficiency. Neonates were allergy to therapeutic drugs or methods.

### 2.2. Therapies

After admission, the two groups of neonates were treated with 21%-80% oxygen concentration, 6-8 L/min gas flow rate, and 4-7 CMH pressure. When CPAP decreased to 2-3 cmH_2_O and oxygen concentration decreased to 25%, dyspnea was significantly relieved or disappeared; the treatment was terminated. If the oxygen concentration was >80%, the pressure was >6-7 cmH_2_O, and the oxygen saturation was still <85% after 6-8 hours of treatment, or type II respiratory failure occurred, the treatment method was changed to mechanical ventilation. On the basis of the above, neonates in the observation group were injected with exogenous PS [17] into trachea as soon as possible.

### 2.3. Sample Collection and ELISA Detection

After the patient was admitted to hospital and at 7: 00 a.m. the next morning after treatment, 5 mL of sterile venous blood was collected and loaded into the coagulation tube. The serum was collected by centrifuge (3000 x g at 4°C for 10 min) and stored in the refrigerator at -80°C. The levels of KRT-14 and ET-1 were detected by ELISA. Blank well, standard sample well, and sample to be tested well were set up. S0 standard substance with the concentration of 0 was added into the blank well, and 50 *μ*L of standard substance with different concentrations was added to the standard well. In the sample well, 10 *μ*L of sample to be tested was firstly added to it and then added with sample diluent 40 *μ*L. Nothing was added to the blank well. In addition to the blank wells, 100 *μ*L of HRP labeled detection antibody was added to each of the standard wells and the sample wells. The reaction wells were sealed with a sealing plate membrane and incubated in a water bath at 37°C for 65 min. The liquid was discarded, and the absorbent paper was patted dry. Each well was filled with washing liquid and allowed to stand for 2 min. The washing liquid was thrown off, and the absorbent paper was patted dry. This procedure was repeated 6 times. Substrates A and B were added to each well, 50 *μ*L each, and incubated at 37°C in the dark for 10 min. The OD value of each well was measured at 450 nm wavelength within 15 min after adding 50 *μ*L of stop solution to each well. Calculate the concentration.

RETRACTED

### 2.4. Efficacy Evaluation

For effective, after treatment, the clinical symptoms of the neonates disappeared or relieved, X-ray films showed that abnormal shadow areas of the lungs disappeared or improved, and blood gas indexes were normal or improved. For ineffective, after treatment, the clinical symptoms of the neonates became worse or did not improve or even died, X-ray films showed enlarged or not improved shadow areas, and blood gas indexes deteriorated or did not improve.

### 2.5. Outcome Measures

For main outcome measures, the expression of KRT-14 and ET-1 in the observation group and the control group was compared, and the therapeutic effect, death, and complications of the two groups were compared.

For secondary outcome measures, the clinical data of the two groups of neonates were compared. The blood gas indexes PaO_2_, PaO_2_, and PaO_2_/FiO_2_ of the two groups of neonates were compared. The diagnostic value of KRT-14 and ET-1 in the therapeutic effect of NRDS neonates was analyzed by using receiver operating characteristic curve (ROC).

### 2.6. Statistical Analysis

SPSS20.0 (SPSS, Chicago, USA) was utilized to carry out statistical analysis on the collected data. GraphPad Prism 7 (GraphPad, San Diego, USA) was adopted for pictures drawing of the collected data. Enumeration data were expressed as (%), qualified by chi-square test, and expressed by x2. Measurement data were expressed by mean standard deviation (Means ± SD). All measurement data were in accordance with normal distribution. Independent sample *t*-test was used for comparison between the two groups. ROC was used to evaluate the diagnostic value of KRT-14 and ET-1 in the therapeutic effect of NRDS neonates. *p* < 0.05 was regarded as statistically significant.

RETRACTED

## 3. Results

### 3.1. Clinical Data

By comparing the clinical data of the two groups of neonates, we found that there was no remarkable difference between the two groups in gender, gestational age, body mass, Apgar score, age of pregnant women, hypertension of pregnant women, diabetes of pregnant women, premature rupture of membranes, delivery mode, premature delivery, and delivery history, as shown in Table 1.

Comparison of therapeutic effects and adverse reactions between the two groups

We observed and compared the therapeutic effects of the two groups of neonates after treatment. It was found that the effective rate of the observation group was considerably higher than that of the control group. There was no remarkable difference between the two groups in death, bronchial dysplasia, cyanosis, and shortness of breath, as shown in Table 2.

### 3.2. Blood Gas Index of Two Groups

By comparing the blood gas indexes PaO_2_, PaCO_2_, and PaO_2_/FiO_2_ before and after treatment, we found that there was no remarkable difference between the observation group and the control group in the three before treatment. After treatment, PaO_2_ and PaO_2_/FiO_2_ in both groups were notably higher than before treatment, while PaCO_2_ was notably lower than before treatment. The levels of PaO_2_ and PaO_2_/FiO_2_ in the observation group were considerably higher than the control group, while PaCO_2_ was considerably lower than the control group, as shown in Figure 1.

Changes and contents of krt-14 and ET-1 before and after treatment

Comparison of the levels of KRT-14 and ET-1 before and after treatment in the two groups revealed that the levels of them in the observation group were not considerably different from those in the control group before treatment. After treatment, the levels of the two in both groups were notably lower than those before treatment, and the levels of the two in the observation group were considerably lower than those in the control group, as shown in Figure 2.

### 3.3. Diagnostic Value of Therapeutic Effects of KRT-14 and ET-1

By comparing the levels of KRT-14 and ET-1 in neonates with effective and ineffective curative effects, we found that the levels of the two in neonates with ineffective curative effects were considerably higher than those in neonates with effective curative effects (*p* < 0.05). Through ROC, we detected the diagnostic value of KRT-14 and ET-1 in the curative effects of NRDS neonates and found that the area under the curve (AUC) of KRT-14 was 0.791, and the AUC of ET-1 was 0.816, as shown in Table 3 and Figure 3.

RETRACTED

## 4. Discussion

The basic pathogenesis of NRDS is acute diffuse alveolar capillary injury, which leads to increase pulmonary capillary permeability, alveolar, and interstitial edema and ultimately gives rise to type II alveolar cells damage. This kind of damage will reduce pulmonary surfactant, thus leading to a decrease in alveolar surface tension, contraction of alveolar groups, and abnormal pulmonary ventilation/blood flow ratio, eventually triggering severe hypoxemia [18, 19]. Noninvasive positive pressure ventilation can relax the alveoli of neonates, improve the compliance of neonates' lungs, maintain the pressure in alveoli, and keep smooth breathing of neonates. Exogenous PS can supplement the lack of PS in neonates, thus reducing the tension of alveoli in neonates, preventing alveoli atrophy, improving lung respiratory function and lung compliance, and increasing blood oxygen saturation in NRDS, thus to reduce the mechanical ventilation time of neonates [20, 21].

First of all, we compared the therapeutic effect and adverse reactions of the two groups after treatment and found that the therapeutic effect of PS combined with noninvasive positive pressure ventilation was much better than that of noninvasive positive pressure ventilation alone, but there was no statistical difference in mortality rate between the two groups. Then, we compared the blood gas indexes PaO_2_, PaO_2_, and PaO_2_/FiO_2_ of the two groups before and after treatment. After treatment, PaO_2_ and PaO_2_/FiO_2_ increased in both groups, and PaCO_2_ decreased significantly. After treatment, the levels of PaO_2_ and PaO_2_/FiO_2_ in the observation group were remarkably higher than those in the control group, while PaO_2_ was remarkably lower than that in the control group. The blood gas status of NRDS neonates will be remarkably worse than that of normal newborns due to the oxygenation status of the lungs and the respiratory function of the neonates. Once the symptoms of the neonates are controlled and the pulmonary function and respiratory function are improved, the blood gas index of the neonates will return to normal [22]. This also shows that the combined treatment is more effective.

Then, we detected the levels of KRT-14 and ET-1 of neonates in both groups. KRT-14 and ET-1 are two factors related to lung tissue [23, 24]. We found that the levels of KRT-14 and ET-1 in the two groups after treatment were notably lower than those before treatment, and the levels of the two in the observation group after treatment were notably lower than those in the control group. Moreover, we also found that KRT-14 and ET-1 in neonates with ineffective therapeutic effects were remarkably higher than those in neonates with effective therapeutic effects, which further suggests that KRT-14 and ET-1 may be used as therapeutic diagnostic indicators for NRDS neonates. Therefore, we evaluated the diagnostic value of therapeutic effect of KRT-14 and ET-1 by ROC and found that the AUC of KRT-14 was, specificity and sensitivity was, and the AUC of ET-1 curve was, specificity and sensitivity was. Both of them have certain diagnostic value in the diagnosis of curative effect of NRDS neonates and may become the diagnostic index of curative effect of potential NRDS neonates.

RETRACTED

However, there are still some deficiencies in our study. The subjects included in our study are all sick neonates, and healthy newborns are not included for comparison. We did not explore differences between the measures tested in this study and healthy newborns. Secondly, there are different types of PS available for treatment [25, 26], so it is hoped that corresponding research can be added in the follow-up for the differences in therapeutic effects of different PS. At last, we found that some complications occurred in the treatment of neonates, but we did not explore the risk factors of these complications. We hope to supplement the corresponding discussion in the follow-up study to improve our point of view.

## 5. Conclusion

PS combined with noninvasive positive pressure ventilation can significantly improve the therapeutic effect of NRDS. KRT-14 and ET-1 levels may be potential therapeutic diagnostic indicators.

## Figures and Tables

**Figure 1:** Changes of blood gas indexes before and after treatment. (a) There was no significant difference in PaO_2_ between the observation group (42.39 ± 6.14) and the control group (41.01 ± 5.89) (*t* = 1.338, *p* = 0.183). PaO_2_ in both groups was significantly increased after treatment (*p* < 0.05), and it in the observation group (76.92 ± 5.94) was significantly higher than the control group (68.54 ± 5.96) (*t* = 8.226, *p* < 0.001). (b) There was no significant difference in PaCO_2_ between the observation group (51.38 ± 4.57) and the control group (52.64 ± 3.89) (*t* = 1.725, *p* = 0.087). PaCO_2_ in both groups was significantly decreased after treatment (*p* < 0.05), and it in the observation group (35.58 ± 3.10) was significantly lower than the control group (43.08 ± 3.83) (*t* = 12.659, *p* < 0.001). (b) There was no significant difference in PaO_2_/FiO_2_ between the observation group (189.19 ± 10.95) and the control group (192.05 ± 11.55) (*t* = 1.487, *p* = 0.139). PaO_2_/FiO_2_ in both groups was significantly increased after treatment (*p* < 0.05), and it in the observation group (426.97 ± 41.39) was significantly higher than the control group (387.18 ± 28.86) (*t* = 6.115, *p* < 0.001). ^∗∗^ denotes *p* < 0.01; ^∗∗∗^ denotes *p* < 0.001.

RETRACTED

**Figure 2:** Levels of KRT-14 and ET-1 before and after treatment. (a) There was no significant difference in KRT-14 between the observation group (4.38 ± 0.84) and the control group (4.41 ± 0.70) (*t* = 0.822, *p* = 0.225). KRT-14 in both groups was significantly decreased after treatment (*p* < 0.05), and it in the observation group (2.99 ± 0.64) was significantly lower than the control group (3.31 ± 0.51) (*t* = 3.206, *p* < 0.002). (b) There was no significant difference in ET-1 between the observation group (51.34 ± 5.13) and the control group (49.90 ± 4.75) (*t* = 1.697, *p* = 0.092). ET-1 in both groups was significantly decreased after treatment (*p* < 0.05), and it in the observation group (33.29 ± 3.93) was significantly lower than the control group (41.51 ± 4.48) (*t* = 11.441, *p* < 0.001). ^∗∗∗^ denotes *p* < 0.001.

**Figure 3:** Diagnostic value of curative effect of KRTt-14 and ET-1. (a) KRT-14 in neonates with effective therapeutic effect (2.94 ± 0.56) was significantly lower than that in neonates with ineffective efficacy (3.70 ± 0.65) (*t* = 5.472, *p* < 0.001). (b) ET-1 in neonates with effective therapeutic effect (33.80 ± 5.36) was significantly lower than that in neonates with ineffective efficacy (42.68 ± 4.48) (*t* = 6.997, *p* < 0.001). (c) ROC of KRT-14 in diagnosis of therapeutic effect after treatment. (d) ROC of ET-1 in diagnosis of therapeutic effect after treatment. ^∗∗∗^ denotes *p* < 0.001.

**Table 1:** Clinical data.

	Observation group (*n* = 73)	Control group (*n* = 64)	*X* ^2^/*t*	*p*
Gender				
Male	38 (52.05)	37 (57.81)		
Female	35 (47.95)	27 (42.19)	0.456	0.499
Gestational age (weeks)	33.37 ± 2.12	32.87 ± 2.05	1.399	0.164
Body mass (kg)	2.82 ± 0.69	2.71 ± 0.58	1.002	0.318
Apgar score	8.47 ± 1.31	8.28 ± 1.26	0.862	0.390
Age of pregnant woman (years)	27.3 ± 4.8	26.5 ± 4.1	1.041	0.230
Hypertension of pregnant women	9 (12.33)	5 (7.81)	0.758	0.384
Diabetes of pregnant women	11 (15.07)	7 (10.94)	0.510	0.475
Premature rupture of membranes	9 (12.33)	10 (15.63)	0.310	0.578
Delivery mode				
Eutocia	41 (56.16)	40 (62.50)	0.566	0.452
Cesarean section	32 (43.84)	24 (37.50)		
Premature delivery				
Yes	52 (71.23)	41 (64.06)	0.804	0.370
No	21 (28.77)	23 (35.94)		
Delivery history			0.027	0.870
Primiparity	50 (68.49)	43 (67.19)		
Multiparity	23 (31.51)	21 (32.81)		

RETRACTED

**Table 2:** Therapeutic effect and adverse reactions.

	Observation group (*n* = 73)	Control group (*n* = 64)	*t*	*p*
Effective curative effect	67 (91.78)	51 (79.69)	4.175	0.041
Ineffective curative effect	6 (8.22)	13 (20.31)		
Death	3 (4.11)	6 (9.38)	1.540	0.215
Bronchial dysplasia	6 (8.22)	11 (17.19)	2.514	0.112
Cyanopathy	8 (10.96)	10 (15.63)	0.651	0.420
Shortness of breath	9 (12.33)	14 (21.88)	2.225	0.136

**Table 3:** ROC.

Index	AUC	95% CI	Specificity	Sensitivity	Youden index	Cut-off
KRT-14	0.791	0.665~0.917	85.47%	60.00%	45.47%	>3.645
ET-1	0.816	0.726~0.907	76.07%	70.00%	46.07%	>40.060

## Data Availability

The datasets used and/or analyzed during the current study are available from the corresponding author on reasonable request.
